This article has been retracted.

# Cancer-Associated Fibroblasts-Derived Exosomes Suppress Immune Cell Function in Breast Cancer via the miR-92/PD-L1 Pathway

**DOI:** 10.3389/fimmu.2020.02026

**Published:** 2020-10-09

**Authors:** Dongwei Dou, Xiaoyang Ren, Mingli Han, Xiaodong Xu, Xin Ge, Yuanting Gu, Xinxing Wang

**Affiliations:** ^1^Department of Breast Surgery, The First Affiliated Hospital of Zhengzhou University, Zhengzhou, China; ^2^Department of Information, The First Affiliated Hospital of Zhengzhou University, Zhengzhou, China

**Keywords:** YAP1, miR-92, PD-L1, CAF, breast cancer

## Abstract

Cancer-associated fibroblasts (CAFs) are an essential component in the tumor microenvironment and have been reported to contribute to tumor progression through many mechanisms; however, the detailed mechanism underlying the immune-suppression effect of CAFs is not clearly defined. In this study, human breast cancer-derived CAFs were cultured, and CAF-derived exosomes in a culture medium were isolated. Using a miRNA profiles assay, we identify a significantly higher level of microRNA-92 isolated in CAFs exosomes. After treatment by CAF-derived exosomes, breast cancer cells express higher programmed cell death receptor ligand 1 (PD-L1), accompanied with increased miR-92 expression. Increased PD-L1 expression, which was induced by CAF-derived exosomes, significantly promotes apoptosis and impaired proliferation of T cells. The underlying mechanism of this effect was studied, proliferation and migration of breast cancer cells were increased after the transfection of miR-92, LATS2 was recognized as a target gene of miR-92, and further confirmed by a luciferase assay. Immunoprecipitation showed that LATS2 can interact with YAP1, chromatin immunoprecipitation confirmed that after nuclear translocation YAP1 could bind to the enhancer region of PD-L1 to promotes transcription activity. Furthermore, the animal study confirmed that CAFs significantly promoted tumor progression and impaired the function of tumor-infiltrated immune cells *in vivo*. Our data revealed a novel mechanism that can induce immune suppression in the tumor microenvironment.

## Introduction

Breast cancer is the second most common cancer worldwide, the fifth most common cause of cancer death, and the leading cause of cancer death in women (1, 2).

A high expression of the programmed cell death receptor ligand 1 (PD-L1) was associated with poor prognosis in breast cancer (3, 4). Cancer-associated fibroblasts (CAFs) are one of the most important components in the tumor microenvironment of breast cancer; it was reported that CAFs can support the progression of breast cancer through many mechanisms, and promotes migration and proliferation of cancer cells (5–7). Recently, several studies have shown that CAFs also can suppress the immune response in the tumor microenvironment by recruiting M2 macrophages or directly suppressing the function of immune cells (8–10). Cancer-associated fibroblasts can affect other cells within the tumor microenvironment by secreting growth factors, cytokines, and exosomes, and it is well documented that CAFs can interact with tumor cells by exosomes (11). Exosomes are small vesicles with a diameter ranging from 40 to 100 nm. The exosomes derived from endocytic compartments can contain RNA, protein, DNA, and microRNA (12).

microRNAs are evolutionarily conserved class of 22-nucleotide non-coding RNAs. microRNA can negatively regulate target gene expression in a sequence-specific manner and has been reported to play an important role in metabolism, migration, and apoptosis of cancer cells (13–16).

To date, the effect of breast cancer CAF-derived exosomes on immune cells has not been studied. In this study, we found that CAF-derived exosomes can significantly promote PD-L1 expression in breast cancer cells and subsequently induce the apoptosis of T cells and impair NK cells function. Mechanically, it is observed that after treatment with CAF-derived exosomes, miR-92 expression in breast cancer cells was increased significantly, as the target gene of miR-92, LATS2, was downregulated, which subsequently enhanced the nuclear translocation of YAP1. YAP1 binds to the enhancer region of PD-L1, and enhances PD-L1 transcription activity. Further, the immune suppression effect was also confirmed *in vivo*, which showed that CAFs can suppress immune cell function.

Overall, this study revealed a novel mechanism that can induce immune suppression in the tumor microenvironment.

## Results

### Cancer Associated Fibroblast-Derived Exosomes Promote miR-92 and PD-L1 Expression in Breast Cancer

Breast CAFs were isolated and cultured, as shown in Figure 1A, the immunofluorescence shows that CAFs were positive for fibroblast-specific protein 1 (FSP) and vimentin, to further confirm the phenotype of CAFs, western blot was performed. As shown in Figure 1B, CAFs express higher FSP, vimentin, and α-SMA compared with normal fibroblasts (NFs), which were isolated from para-cancer normal tissue. These data indicated that we had isolated breast cancer-derived CAFs successfully. Then CAF-derived exosomes were isolated and, as shown in Figures 1C,D, purified. Exosomes from the condition medium of CAFs displayed typical morphology and size, and contained exosomes markers CD63, CD9, and ALIX (Figure 1E). miRNA expression profiles of CAF-derived exosomes and NF-derived exosomes were examined, as mentioned in the materials and methods, the expressions of 2026 human miRNAs were analyzed by using a SYBR Green-based real-time PCR array. We found that 16 and 45 miRNAs were significantly (*P* < 0.01) upregulated and downregulated in CAF-derived exosomes, respectively, compared to those of NF exosomes. As shown in Figure 1F, the top five most upregulated miRNA in CAF-derived exosomes were hsa-miR-92, hsa-miR-7854, hsa-miR-513c, hsa-miR-544b, and hsa-miR-3161.

**FIGURE 1:** Cancer associated fibroblast-derived exosomes promote miR-92 and PD-L1 expression in breast cancer. **(A)** Immunofluorescence image of FSP and vimentin in breast cancer-derived cancer associated fibroblasts. **(B)** Western blot analysis of FSP, vimentin, α-SMA expression in cancer-associated fibroblasts and normal fibroblasts. **(C)** Transmission electron microscopy image of exosomes. **(D)** TRPS analysis of exosomes confirming the expected size range of 30–150 nm in diameter. **(E)** Western blot analysis of exosome markers in CAF-derived exosomes and cell lysates. **(F)** A clustergram performed hierarchical clustering of the upregulated and downregulated miRNAs in exosomes isolated from CAFs compared with normal fibroblasts cells. The data display a heat map with an indication of co-regulated genes across groups or individual samples. The magnitude of gene expression is presented by colors as indicated by the color bar shown on the right. **(G)** micro-RNA expression after exosomes treatment **(H)** flow cytometry analysis of PD-L1 expression in breast cancer cells. **(I)** PD-L1 expression analyzed by Western blot. Error bars represent mean ± SD; ****P < 0.0001; n.s., not significant; by paired two-sided Student’s *t*-test.

To confirmed whether upregulated miRNA in exosomes subsequently influences miRNA expression in tumor cells, real-time PCR was performed, as shown in Figure 1G. After the breast cancer cell line MCF7 was cultured with CAF-derived exosomes, no significant alternation in selected miRNA expression was observed except for miR-92, which upregulated significantly after exosome treatment. Moreover, we also found PD-L1 expression in cancer cells increased after being treated with CAF-derived exosomes (Figure 1H). This was further confirmed by Western blot (Figure 1I).

### miR-92 Promotes Migration and Proliferation of Breast Cancer Cells

Based on previous results, we were curious about the role played by miR-92 in breast cancer. As shown in Figure 2A, the clinical sample showed that breast cancer tissue expresses higher miR-92 compared with normal tissue, implying a possible tumor-promotion role played by miR-92. Breast cancer cells MCF7 were transfected with a mimic and inhibitor of miR-92, the efficiency of transfection was confirmed by real-time PCR (Figure 2B). A CCK-8 and colony genesis experiment showed that after the upregulation of miR-92, MCF7 presented a higher proliferation rate compared with negative control (Figures 2C,D), and the downregulation of miR-92 inhibited MCF7 proliferation. A wound-healing assay showed that miR-92 promotes migration, and the downregulation of miR-92 inhibited the migration of breast cancer cells, this effect was further confirmed by a Transwell assay (Figure 2E,F). Taken together, our results indicated that miR-92 promotes migration and proliferation of breast cancer cells.

**FIGURE 2:** miR-92 promotes migration and proliferation of breast cancer cells. **(A)** miR-92 expression was examined by qRT-PCR in human breast cancer tissue and normal tissue. In total, 32 cancer tissues and 34 normal tissues were analyzed. **(B)** miR-92 expression after transfection of miR-92 mimic or inhibitor was analyzed by qRT-PCR (*n* = 3). **(C)** miR-92 overexpression promotes cell proliferation. Cancer cells were transfected with a miR-92 mimic or inhibitor and the absorption (A450 nm) was detected at 0, 24, 48, and 72 h, respectively. **(D)** Cancer cells transfected with the miR-92 mimic and NC control were assayed for clonogenicity in adherent cultures. **(E)** A wound-healing closure assay for cancer cells which transfected with the miR-92 mimic or inhibitor (magnification, ×50, scale bar: 500 μm). **(F)** Transwell assay for cancer cells which transfected with the miR-92 mimic or inhibitor (magnification, ×100). Error bars represent mean ± SD; ****P < 0.0001; n.s., not significant; by paired two-sided Student’s *t*-test.

### miR-92 Targeting LATS2 and Enhance Nuclear Translocation of YAP1

To find out the target gene for miR-92, bioinformation screening using the TargetScan database was performed. Based on the database, LATS2 may serve as a target protein of miR-92. A luciferase report assay was used to confirm the direct target for miR-92, as shown in Figure 3A. Wild-type LATS2 3’-UTR and mutant LATS2 3’-UTR with a nucleotide substitution in the putative binding site was subcloned into a luciferase report vector, after co-transfection of the miR-92 mimic, luciferase activity was suppressed, whereas in the luciferase with mutant UTR, this effect was not observed. These data have shown that LATS2 is a direct target of miR-92 in breast cancer cells. To figure out the underlying role played by LATS2 in breast cancer, we investigated LATS2 expression in the GEO dataset, as shown in Figure 3B. LATS2 was upregulated in normal tissue compared with tumor tissue, indicated that LATS2 might be a tumor suppression gene. As shown in Figure 3C, based on gene analysis of STRING, LATS2 possibly interacts with YAP1. To test this possibility, Western blot was performed. As shown in Figure 3D, after LATS2 was downregulated by miR-92 transfection, the phosphating of YAP1 was decreased, and nuclear translocation of YAP1 was increased subsequently, moreover, after LATS2 was upregulated by the transfection of the miR-92 inhibitor, the nuclear translocation of YAP1 was decreased. To further confirm the relationship between YAP1 and LATS2, a co-immunoprecipitation (co-IP) assay was performed. As shown in Figure 3E, it is observed that YAP1 could precipitate with LATS2; these data confirmed that LATS2 could interact with YAP1 directly, LATS2 promotes the phosphating of YAP1 and reduces its nuclear translocation.

**FIGURE 3:** miR-92 targeting LATS2 and enhance nuclear translocation of YAP1. **(A)** Schematic representation of the miR-92 targeting sequences within the 3′UTR of LATS2. A luciferase reporter assay was conducted in MCF7 cells following transfection with the miR-92 mimic or NC, and together with WT or Mut LATS2 3′UTR luciferase reporter plasmid. **(B)** LATS2 expression was examined in normal and breast cancer tissue from a public dataset. **(C)** The protein–protein network view from the STRING database showing the networks of LATS2. **(D)** Western blot shows the YAP1, LATS2 expression in MCF7 which transfected with the miR-92 mimic or inhibitor. **(E)** Co-IP analysis with anti-YAP1 antibody or IgG in MCF7. **(F)** Western blot analysis of YAP expression after two shRNA target YAP was transfected. **(G)** Transwell assay for breast cancer cells which transfected with the miR-92 mimic and/or shRNA targeting YAP (magnification, ×100). Error bars represent mean ± SD; ****P < 0.0001; n.s., not significant; by paired two-sided Student’s *t*-test.

To further confirm the function of YAP1 in the miR-92 induced effect, YAP1 was knocked down by shRNA transfection. The effect of the YAP1 downregulation was confirmed by Western blot (Figure 3F). After YAP1 was knocked down, increased migration capacity induced by miR-92 was partly impaired, indicated that the pro-tumor effect of miR-92 partly relies on the LATS2/YAP1 pathway (Figure 3G).

Collectively, these results have shown that LATS2 is a direct target of miR-92, LATS2 can interact with YAP1 and regulate nuclear translocation of YAP1 in breast cancer cells.

### miR-92 Promotes PD-L1 Transcription Activity by Enhancing the Nuclear Translocation of YAP1

It has been shown that CAF-derived exosome treatment enhances PD-L1 expression in tumor cells, we sought to confirm if upregulation of miR-92 can promote PD-L1 expression, as shown in Figure 4A. Western blot indicated that miR-92 overexpression results in increased YAP1 nuclear translocation, followed by the upregulation of PD-L1. After the expression of LATS2 was enhanced by the transfection of the miR-92 inhibitor, a decreased YAP1 nuclear translocation can be observed, followed by the downregulation of PD-L1. This effect was further confirmed by flow cytometry, as shown in Figure 4B.

**FIGURE 4:** miR-92 promotes PD-L1 transcription activity by enhancing the nuclear translocation of YAP1. **(A)** Western blot shows the YAP1, LATS2, and PD-L1 expression in MCF7 which was transfected with the miR-92 mimic or inhibitor. **(B)** Flow-cytometry analysis for PD-L1 expression in MCF7 which was transfected with NC or miR-92. Blank is an unstained group indicating negative fluorescence intensity. **(C)** ChIP assay was performed with MCF7 which is shown by gel bands of the RT-PCR products with 30 cycle. **(D)** Western blot shows the YAP1 and PD-L1 expression in MCF7 which was transfected with the miR-92 mimic or inhibitor or/and shRNA targeting YAP.

YAP1 is a transcription co-activator and together with the TEAD family protein regulates many genes. To explain the underlying mechanism that causes increased PD-L1 expression after nuclear translocation of YAP1, we hypothesis that YAP1 could promote PD-L1 transcription. A TEAD-binding site was observed in 7911 bps upstream of a PD-L1 transcription start site. Chromatin immunoprecipitation (ChIP) was performed to test this possibility. As shown in Figure 4C, the YAP1 antibody causes precipitation in PD-L1 enhancer regions encompassing the putative TEAD binding site. Although, this was not observed in the ChIP assay using Rabbit IgG; these results confirmed that YAP1 could occupy the enhancer region of PD-L1 directly.

To further confirm whether the occupation of YAP1 in enhancer regions of PD-L1 can result in increased transcription activity of PD-L1, YAP1 was knocked down by the transfection of siRNA, as shown in Figure 4D. After YAP1 was knocked down, nuclear translocation of YAP1 also decreased significantly, as expected, YAP1 downregulation also diminished PD-L1 upregulation which resulted from miR-92 overexpression.

Collectively, our result confirmed that miR-92 can promote PD-L1 expression by enhancing occupation between YAP1 and PD-L1 enhancer regions.

### Exosome-Induced PD-L1 Upregulation Suppresses Immune Cell Function in Breast Cancer

Programmed cell death receptor ligand 1 is a type 1 transmembrane surface glycoprotein encoded by the CD274 gene; it promotes T cell tolerance and escapes host immunity. It can bind to its ligand programmed cell death protein 1 (PD-1), which is usually expressed in immune cells and suppresses the function of immune cells. The expression of PD-1 in NK cells can be induced after NK cells are co-cultured with tumor cells; we asked whether the function of NK cells which express PD-1 can be suppressed by exosomes induced PD-L1 overexpression. To answer this question, the NK cell killing assay was performed, as shown in Figure 5A. PD-1-expression NK cells can lyse cancer cells significantly, but the function of NK cells were impaired when tumor cells were pre-treated by exosomes. The function of NK cells can be partly rescued after the administration of the anti-PD-L1 antibody.

**FIGURE 5:** Exosomes induced PD-L1 upregulation suppresses immune cell function in breast cancer. **(A)** An NK cell cytotoxicity assay was performed, MCF7 treated or untreated by exosomes were used as target cells. The quantification of cytotoxicity of NK cells were shown in right panel. **(B)** CFSE was used to evaluate the proliferation of T cells. T cells were cultured directly with MCF7 treated or untreated by exosomes for 48 h. **(C)** T cells were cultured directly with MCF7 treated or untreated by exosomes for 48 h, the apoptosis rate was evaluated by an Annexin V stain. Error bars represent mean ± SD; ****P < 0.0001; n.s., not significant; by paired two-sided Student’s *t*-test.

PD-1 is classically expressed in T cells, as shown in Figures 5B,C. When T cells were co-cultured with cancer cells which were pre-treated by exosomes, an enhanced apoptosis rate, and impaired proliferation rate was observed. As we expected, those effects can be partly blocked by the administration of the anti-PD-L1 antibody. Importantly, the knocking down of YAP1 markedly reduced exosome-induced apoptosis of T cells indicating that the immune suppression effect of exosomes relied on the expression of YAP1 and PD-L1.

### Cancer-Associated Fibroblasts Promote Tumor Progression and Suppress Immune Cell Function *in vivo*

An animal experiment was performed to investigate the role played by CAFs *in vivo*. Mesenchymal stem cells, which are a precursor of CAFs, were used in this xenograft model. MA-782-mCherry alone and MA-782-mCherry mixed with MSCs were injected into the flanks of Balb/c mice. The mice were sacrificed after three weeks, as shown in Figure 6. An MA-782-mCherry mixed with MSCs generated a larger tumor volume than those produced by MA-782-mCherry alone, and a heavier tumor weight in MA-782-mCherry mixed with MSCs was observed compared with MA-782-mCherry alone. This result indicated that CAFs could promote tumor progression *in vivo*.

**FIGURE 6:** Cancer associated fibroblasts promote tumor progression and suppress immune cell function *in vivo*. **(A)** The weight of tumors isolated from the mice with MA-782 cells co-injected with or without MSC (*n* = 8). **(B)** PD-L1 expression of MA-782 which gated as mCherry+. **(C,D)** CD107a expression of cytotoxicity T cells and NK cells. Error bars represent mean ± SD; ****P < 0.0001; n.s., not significant; by paired two-sided Student’s *t*-test.

To investigate the underlying mechanism responsible for tumor volume, sigle cell suspension of the tumor was analyzed by flow cytometry. As shown in Figure 6B, cancer cells in the tumor which expressed mCherry were studied, PD-L1 in tumor cells, which gated as mCherry+ were examined, the result confirmed that tumor cells express higher PD-L1 *in vivo* after the addition of MSCs. To test the effect of PD-L1 *in vivo*, NK cells and cytotoxic T cells were gated as CD49b+CD335+ and CD8+CD4+, respectively. CD107a (LAMP-1) may be a marker for the degranulation of NK, we used this marker to test the function of immune cells. As shown in Figures 6C,D, the addition of MSCs significantly reduced CD107a expression in NK cells and T cells; the result indicated that CAFs could suppress the function of immune cells *in vivo*.

Taken together, our results indicated that CAFs promote tumor progression and suppress immune cell function *in vivo*.

## Discussion

Breast cancer remains a significant threat to the health and wellness of women in the United States, accounting for 30% of all new cancer diagnoses and almost 41,000 deaths annually (17–19). Immunotherapy is an effective strategy for a variety of cancers and has been shown to promote impressive survival benefits in patients (20–23), however, most breast cancers are resistant to monotherapy with checkpoint inhibitors (24). Cancer-associated fibroblasts are an important component of the tumor microenvironment and have been reported to suppress immune cell function in a variety of tumors, but its underlying mechanism remains unknown. Exosome-based miRNA delivery is one strategy of CAFs to influence other cells present in the microenvironment. In this study, we reported a novel mechanism of immune suppression based on exosomes delivery.

miR-92 has been reported to play an oncogenic role in a variety of cancers (25). In this study, we observed that after the treatment of CAF-derived exosomes, miR-92 expression was significantly increased, whereas other selected micro-RNA expression remained stable. We subsequently investigated the role of miR-92 in breast cancer cells. As previously reported, we found that the upregulation of miR-92 promotes migration and invasion in breast cancer cells.

Programmed cell death receptor ligand 1 is a type 1 transmembrane surface glycoprotein encoded by the CD274 gene, it promotes T cell tolerance and escapes host immunity, but the regulation of PD-L1 in the tumor is still under investigation (26–28). In this study, we used a luciferase activity assay to confirm that LATS2, which is an important component of the Hippo pathway, was a direct target of miR-92. Co-IP was performed to confirm that LATS2 could directly interact with YAP1, LATS2 promotes YAP1 phosphating and subsequently prevents YAP1 nuclear translocation. It has been reported that YAP1 activity can regulate PD-L1 expression in some types of cancer (29, 30). In this study, ChIP was used to confirm that YAP1 directly occupied the enhancer regions of PD-L1, and subsequently resulted in the upregulation of PD-L1.

We further confirmed the immune suppression effect of CAF-derived exosomes and found that after cancer cells were treated by CAF-derived exosomes, co-culture with cancer cells resulted in an increased apoptosis rate and impaired immune cell function.

We further confirmed our proposed mechanism *in vivo*, based on flow cytometry, we confirmed that CAFs significantly suppressed immune cell function *in vivo*, and promoted PD-L1 expression in breast cancer cells.

Collectively, this study revealed a novel mechanism that can induce immune suppression in the tumor microenvironment.

## Materials and Methods

### Ethics Statement

Breast cancer tissues were obtained from patients who had undergone surgery at The First Affiliated Hospital of Zhengzhou University. Written informed consent was obtained from all participants, and all procedures were authorized by the Ethical Committee of The First Affiliated Hospital of Zhengzhou University.

### Antibodies and Reagents and Cell Lines

Anti-LATS2, YAP1, lamin-B, PPD-L1, GAPDH rabbit polyclonal (Abcam, Cambridge, United Kingdom), and anti-actin polyclonal (Santa Cruz Biotechnology) antibodies were used at 1:1,000 dilution for Western blotting. Anti-rabbit polyclonal secondary horseradish peroxidase-conjugated antibodies were used for detection (diluted; 1:2,000). Paclitaxel (TX) was purchased from Sigma (St. Louis, MO). The working stock was diluted in the media at a final concentration of 4μM and further diluted when needed. The human ovarian serous cancer cell line, MCF7 cells were obtained from ATCC (Manassas, VA, United States). These cells were cultured in Dulbecco’s modified Eagle’s medium (DMEM) plus 10% fetal bovine serum (FBS) at 5% CO_2_ and 37°C.

### microRNA Expression Profiling

Total RNA extraction and miRNA expression profiling were performed by QIAGEN (QIAGEN, Hilden, Germany). All exosome samples were packed in tightly sealed vial tubes and shipped with 25 kg of dry ice. Briefly, total RNAs were extracted from 300 μg of CAF-derived exosomes and NF-derived exosomes. cDNA synthesis was performed using the miScript II RT Kit and amplified by the miScript PreAMP PCR Kit. The miRNA expression profiling was performed using the miScript miRNA PCR Array that covers 22026 human miRNAs.

### Wound-Healing and Transwell Assays

For the wound-healing assay, cells were seeded on six-well plates. When 95% confluence was achieved, the cell monolayer was gently scratched using a 200-μm sterile plastic pipette tip. Then, the wound was photographed. After 24 h, the healing wound was photographed. For Transwell migration or invasion assays, 4 × 10^4^ cells suspended in medium without serum were seeded in the upper chamber membranes coated without/with Matrigel (BD Biosciences). Then, a 600 μL medium with 10% FBS was added to the lower chamber. After 24 h, the underside of the membrane was fixed for 30 min and stained with 0.1% crystal violet. The inner side of the membrane was wiped with a cotton swab. Then, cells were quantified under a microscope.

### Detection of NK Cells Killing Activity

NK-92 cells were added into 1 × 10^5^ cancer cells, which were labeled with CFSE and incubated at 37°C for 5 h. After the incubation, all cells were stained with 7-AAD (BD Bioscience). Cells were subsequently analyzed by flow cytometry.

### Transmission Electron Microscopy

For transmission electron microscopy (TEM), 10 μL of exosome suspension was absorbed onto carbon-coated copper grids (200 mesh) for 1 min. Samples were washed with double-distilled water and negatively stained with 2% uranyl acetate solution for 1 min. After being air dried, the samples were visualized at 87,000× in a Phillips Tecnai transmission electron microscope at 80 kV.

### Exosome Size Analysis

Tunable resistive pulse sensing (TRPS) technology was used to investigate the size and numbers of the exosomes. The TRPS apparatus is an iZon-qNano (iZon Science Europe Ltd., Oxford, United Kingdom). The measuring cell used for these experiments is a NP100 membrane (iZon Science Europe Ltd.). The concentration of particles was standardized using multi-pressure calibration with 70 nm carboxylated polystyrene beads at a concentration of 1.5 × 10^11^ particles/mL, as previously reported (31).

### Isolation of Mesenchymal Stem Cells

In brief, bone marrow was collected from the femurs and tibias of 8–10 week-old C57BL/6 or Balb/c male mice. For MSC isolation, the cells were carefully suspended and passed through a 70 mm strainer, spun down, and resuspended in a minimal essential medium supplied with 10% MSC certified FBS (Thermo Fisher Scientific, Waltham, MA, United States) and antibiotic-antimycotic solution (100 units of penicillin, 100 mg of streptomycin, and 0.25 mg of amphotericin B per milliliter, HyClone; Thermo Fisher Scientific). The medium was replaced the next day to remove the unattached cells.

### Flow Cytometry Analysis

Cells were digested with trypsin and then washed by PBS. The Annexin V-FITC Apoptosis Detection Kit (Beyotime) was applied to practice cell apoptosis in line with the manufacturer’s instructions. The apoptotic cells were dual-stained with PI and Annexin V-FITC, using the Annexin V/FITC kit (Thermo Fisher Scientific, Shanghai, China). The analysis was carried out via the BDTM LSRII flow cytometer (BD Biosciences). Afterward, data were measured with the Cell Quest (BD Bioscience, San Jose, CA, United States) software.

### Isolation of Cancer-Associated Fibroblasts and Normal Fibroblasts

CAFs and primary colorectal NFs were isolated from breast cancer tissues and adjacent normal tissue. Briefly, the specimen was cut into sections, then subjected to collagenase IV (Invitrogen, CA, United States) digestion for 3 h at 37°C. After digestion, it was passed through a 70 μm mesh (BD Falcon, CA, United States). We centrifuged the filtrate and cultivated the cells in red blood cell lysis buffer to eliminate red blood cells, washed the remaining cells with PBS. The cells for analysis were re-suspended in FACS staining buffer for flow cytometry, cells for culturing were then plated in DMEM with low glucose content containing 10% FBS (Gibco, United States) and 1% penicillin/streptomycin, adherent cells were removed to other culture dishes for the cultivation of CAFs and NFs. For the collection of CM, 2 × 10^6^ cells were seeded onto a 10-cm plate and cultured for 36 h, the medium was replaced with 5 mL fresh F12 without serum and cells were cultured for a further 24 h, the CM was collected and filtered and stored at −40°C.

### Exosome Preparation and Analysis

Exosomes were collected by Iodixanol Density Gradient Ultracentrifugation according to previously published protocol (32). In brief, the CAFs or NFs were incubated for 48 h in complete PRMI1640 medium with 10% FBS that was previously depleted of contaminating vesicles by overnight centrifugation at 100,000 × *g* using a Beckman Coulter Allegra^®^ X-15R centrifuge. Density gradient ultracentrifugation was performed by loading the sample onto 50, 30, and 10% iodixanol layers and then centrifuged at 120,000 × *g* for 24 h.

### Luciferase Reporter Assay

A luciferase reporter assay was used to test the miR-92/LATS2 relationship. The firefly luciferase reporter gene expression vector, controlled with the SV40 enhancer, was purchased from GeneCopoeia. The wild-type or mutant LATS2 3’-UTR sequence (LATS2; NM_014572; HmiT007288- MT06) was inserted downstream of the luciferase gene, whereas no oligonucleotides were inserted in the control vector. Renilla luciferase was used as a tracking indicator for transfection efficiency. The luciferase activity was measured using a LightSwitch Assay Reagent according to the manufacturer’s instructions (SwitchGear Genomics).

### ChIP Assay

Fragmented chromatin from cancer cells was incubated with anti-IgG (negative control) and anti-YAP. Recruited DNA was subjected to PCR using the primers for distal enhancer regions of PD-L1, and PCR products were electrophoresed in agarose gel. The ChIP assay was conducted using the ChIP Assay Kit (Millipore Corporation). Polyclonal antibodies for YAP (Cell Signaling Technology) and control rabbit antibody for IgG (Cell Signaling Technology) were used for ChIP. Primers were used for RT-PCR to amplify the PD-L1 gene.

### Cell Viability Assay

Cell viability was determined by CCK8 assays. Briefly, cancer cells were seeded in 96-well plates (5 × 10^3^ cells/well) and treated with corresponding processes. CCK8 was added into the wells for 3 h at indicated times. The absorbance in each well at a wavelength of 450 nm (A450) was measured with a Thermomax microplate reader.

### Western Blot Analysis and Immunoprecipitation

Cancer cells were collected, washed twice with cold PBS and lysed in NP-40 lysis buffer for 30 min at 4°C. The protein concentration was measured using a bicinchoninic acid assay kit (Thermo). Protein extracts were separated by electrophoresis in an 8–12% premade sodium dodecyl sulfate-polyacrylamide mini gel (Tris-HCL SDS-PAGE) and transferred to a PVDF membrane. The membrane was incubated with indicated antibodies and detected by using a chemiluminescence method. For immunoprecipitation (IP), total cell lysates were incubated with appropriate antibodies overnight and subsequently rotated with protein A/G beads for 2–4 h at 4°C. Beads were washed three times using NP-40 lysis buffer, mixed with 2 × SDS sample buffer, and boiled for 5–10 min. The co-precipitates were analyzed by Western blot analysis.

### Animal Experiment

Animal assays were performed according to the Experimental Animal Care Guidelines. Approximately 6–7 week-old BALB/c mice were bred under specific pathogen-free (SPF) conditions. The mice were divided into four randomized groups (*n* = 6 per group), 1 × 10^5^ CT-26-mCherry with or without BALB/c derived BM-MSC were subcutaneously injected into the flank of each mouse. The tumor size was measured using digital Vernier calipers every 3 days, the tumor volume was calculated as the following formula: volume = 1/2 × (width^2^ × length). All mice were sacrificed after 18 days, and the tumors were collected and visually examined. Then the tumor was cut into sections and subjected to collagenase IV (Invitrogen, CA, United States) digestion for 3 h at 37°C. After digestion, it was passed through a 70 μm mesh (Miltenyi Biotech, Germany) and analyzed by flow cytometry.

### Statistical Analysis

All the data were presented as the mean ± SEM. One-way analysis of variance (ANOVA) was adopted to analyze the differences among groups by using SPSS 13.0 (SPSS Inc., Chicago, IL, United States). Pair-wise comparisons were also made between groups using the Student–Newman–Kuels (SNK) test. A *P*-value of less than 0.05 was considered as statistically significant.

## Data Availability Statement

The raw data supporting the conclusions of this article will be made available by the authors, without undue reservation, to any qualified researcher.

## Ethics Statement

The animal study was reviewed and approved by The First Affiliated Hospital of Zhengzhou University.

## Author Contributions

DD and XW conceived and designed the study. DD and XR did the main experiment. MH analyzed and interpreted the data. XX was responsible for reagents and materials. XG drafted the article. YG and XW revised the article critically. All authors had final approval of the submitted version.

## Conflict of Interest

The authors declare that the research was conducted in the absence of any commercial or financial relationships that could be construed as a potential conflict of interest.
